# Baicalin Ameliorates Radiation-Induced Lung Injury by Inhibiting the CysLTs/CysLT1 Signaling Pathway

**DOI:** 10.1155/2022/2765354

**Published:** 2022-06-24

**Authors:** Wu-An Bao, Yue-Zhen Wang, Xiang Zhu, Juan Lin, Ju-Fen Fan, Yang Yang, Xia Zhou

**Affiliations:** ^1^Department of Radiation Therapy, Cancer Hospital of the University of Chinese Academy of Sciences (Zhejiang Cancer Hospital), Hangzhou, Zhejiang Province, China; ^2^Institute of Cancer and Basic Medicine (IBMC), Chinese Academy of Sciences, Hangzhou, Zhejiang Province, China

## Abstract

**Objective:**

Radiation-induced lung injury (RILI) is a common complication of radiotherapy for thoracic tumors. This study investigated the alleviating effect of baicalin (BA) on RILI and its possible mechanism.

**Methods:**

RILI model was established by chest irradiation (IR) of C57BL/6 mice for 16 weeks. Different concentrations of BA were administered, and dexamethasone (DXM) was used as a positive control. Then, the lung pathological changes were observed by HE and Masson staining. The levels of TGF-*β*, TNF-*α*, IL-1*β*, IL-6, CysLT, LTC4, and LTE4 were measured by ELISA. The CysLT1 expression was detected by qPCR, immunohistochemistry, and western blot. Type II AEC cells were pretreated with LTD-4 to establish the RILI cell model and intervened with different concentrations of BA. Then, the collagen I protein level was measured by ELISA. The CysLT1 and *α*-SMA expression were detected by qPCR, immunofluorescence, and western blot.

**Results:**

BA could effectively improve lung histopathological changes and pulmonary fibrosis. *In vivo*, BA could inhibit the levels of TGF-*β*, TNF-*α*, IL-1*β*, and IL-6 and reduce the levels of CysLT, LTC4, and LTE4. *In vitro*, different concentrations of LTD4 could reduce the viability of type II AEC cells, which could be reversed by the administration of different concentrations of BA. In addition, BA could reduce CysLT1 mRNA, as well as CysLT1 and *α*-SMA protein levels *in vitro* and *in vivo*.

**Conclusion:**

BA attenuated lung inflammation and pulmonary fibrosis by inhibiting the CysLTs/CysLT1 pathway, thereby protecting against RILI.

## 1. Background

Radiation-induced lung injury (RILI) is a common and serious complication of radiation therapy for various tumors and occurs in the early stages of radiation therapy [1, 2]. RILI was divided into two stages: radiation pneumonia in the early stage and radiation lung fibrosis in the later stages [3]. The incidence rate of RILI has reached as high as 20% [4]. The main clinical manifestations of RILI are inflammatory infiltration of alveolar interstitial material, progressive dyspnea, deterioration of lung function, and eventually respiratory failure [5]. At present, RILI was mainly treated from the perspective of anti-inflammatory by glucocorticoid therapy, anti-oxidant therapy, and other methods [6]. There is still a lack of effective treatments for RILI. Thus, it is crucial to investigate the treatment and prevention of RILI.

The cysteinyl leukotrienes (CysLTs) are important inflammatory mediators including LTC4, LTD4, and LTE4 [7]. CysLTs exert their effects mainly by activating type 1 and type 2 CysLT receptors (CysLT1 and CysLT2) [8]. Thompson-Souza et al. found that CysLTs played a vital part in pulmonary inflammation [9]. The representative CysLT is implicated in promoting lung inflammation and remodelling in allergic asthma [10]. Furthermore, it has been shown that CysLT1 antagonists have a therapeutic effect on the lungs [11]. The expression of the CysLT1 receptor in the bronchial mucosa of patients with COPD exacerbation was higher than that of normal subjects or patients with stable COPD [12]. Shimbori et al. investigated the pathogenesis of leukotrienes (LTs) in silica-induced pulmonary fibrosis in mice and found that the CysLTs promoted the progression from acute to chronic pulmonary fibrosis [13]. However, the effect of CysLTs on RILI remains still unclear.

Baicalin (BA) is a flavonoid derived from the roots of *Scutellaria baicalensis* Georgi, which has antibacterial, anti-inflammatory, anti-oxidant, anti-cancer, and other pharmacological functions [14]. BA can relieve lung injury and also plays an important role in clinical practice [15]. BA was found to exert anti-inflammatory and neuroprotective effects by downregulating 5-LOX/CysLT [16]. Furthermore, studies have reported that BA can improve pulmonary fibrosis and pulmonary inflammation [17], and BA also could improve LPS-induced acute lung injury in mice [18]. However, whether BA could ameliorate RILI by the CysLTs/CysLT1 signaling pathway remains unclear, which required us to further explore.

Therefore, based on the establishment of the RILI mouse model and the RILI cell model, this study explored whether BA could improve RILI by inhibiting CysLTs/CysLT1 signaling pathway, thereby further providing new ideas and a theoretical basis for the treatment of RILI.

## 2. Material and Methods

### 2.1. Experimental Animal Grouping and Model Establishment

Thirty-six SPF grade female C57BL/6 mice (8 weeks, 18–20 g) were purchased from Shanghai Slack Laboratory Animal Co. Ltd. (production license No: SCXK (Hu) 2017-0005). The mice were randomly divided into six groups (*n* = 6): control, IR (irradiation), IR + BA 50 mg/kg, IR + BA 100 mg/kg, IR + BA 200 mg/kg, and IR + DXM (dexamethasone).

The RILI animal model was established according to Klein et al. [19]. The mice were anesthetized with pentobarbital sodium, followed by right whole chest IR with _60_Co as the IR source (once a day, each IR was 15 Gy, dose rate 0.5 Gy/min). The control group was treated in the same manner but without IR. The IR + BA 50 mg/kg, IR + BA 100 mg/kg, and IR + BA 200 mg/kg groups were intraperitoneally injected with BA of 50, 100, and 200 mg/kg, respectively. The IR + DXM group was intraperitoneally injected with DXM 1.52 mg/kg. The control and IR groups were administered intraperitoneally with the same normal saline. After 16 weeks of IR treatment, the mice were euthanized. The bronchoalveolar lavage fluids (BALFs), lung tissue, and blood were collected; then the blood and BALFs were centrifuged and the BALFs supernatant, lung, and serum were stored at −80°C.

### 2.2. Type II AEC Cell Culture

The blood in the lungs was firstly flushed (vascular perfusion), and DNaseI (Sigma, St. Louis, MO, USA) solution (250 *μ*g/mL) was instilled into the lungs. The lung tissue was cut into small pieces and digested with 0.25% trypsin at 37°C for 30 min, and then the obtained suspension was filtered and centrifuged, and primary culture was carried out in 25% FBS [20]. Resuspended in medium supplemented with 20% FBS (Zhejiang Tianhang Biotechnology Co. Ltd., 11011-8615) and inoculated into flasks precoated with mouse IgG (Sigma). Nonadherent cells were collected and then centrifuged and resuspended in DMEM with FBS. After 36 h, cell purity was detected by NBT/5-BCIP, and type II AEC cells with a purity of more than 90% were retained.

### 2.3. CCK8 Assay

Stock solutions of 10^−4^ mol/L LTD4 and 10^−3^ mol/L BA were prepared and stored at −70°C. Firstly, type II AEC cells were seeded in 96-well plates, and different concentrations of LTD4 (37.5, 75, 150, and 300 nM) were added and cultured [21]. Afterward, the medium was changed and incubated for 2 h, and the optical density was recorded at 450 nm. The concentration of LTD4 that could have a significant effect on type II AEC cells was determined. Then, type II AEC cells were pretreated with different concentrations of BA (10, 20, 40, and 80 *μ*g/mL) for 2 h and then cotreated with LTD4 for 24 h. Finally, 3 effective concentrations were selected to detect the cell effect, and the time-effect relationship was observed.

### 2.4. HE Staining and Masson Staining

Lung tissues were placed in 10% formalin solution and dehydrated by gradient ethanol, embedded and cut 5 *μ*m sections for HE and Masson staining, respectively. The structural changes in lung tissue and pulmonary fibrosis were observed. The result of HE staining was scored by 2 experts and divided into 5 grades [22], of which 0 was normal; 1 was no epithelial cell swelling and detachment, with only a small amount of inflammatory cell infiltration; 2 was a small amount of epithelial cell swelling and detachment, with significant inflammatory cell infiltration; 3 was a large amount of epithelial cell swelling and detachment accompanied by significant inflammatory cell infiltration; and 4 was a large amount of epithelial cell swelling and detachment and inflammatory cell infiltration.

### 2.5. ELISA Assay

The level of TGF-*β* (Shanghai Enzyme Linked Immunology Co. Ltd., ml057830), TNF-*α* (Jiangsu Enzyme Immunoassay Industrial Co. Ltd., MM-0132M2), IL-1*β* (Jiangsu Enzyme Immunoassay Industrial Co. Ltd., MM-0040M2), and IL-6 (Jiangsu Enzyme Immunoassay Industrial Co. Ltd., MM-0163M2), CysLT (Cayman, Cay500390-96S), LTC4 (Shanghai Enzyme-linked Biotechnology Co. Ltd., ml001970), and LTE4 (Cayman, Cay501060-96S) were detected according to ELISA kits. Type II AEC cells were centrifuged (3,500 r/min, 15 min), and the supernatant was taken to test the content of collagen I protein (Cayman, Cay500390-96S) according to the ELISA kit.

### 2.6. Immunohistochemistry Assay

The lower lobes of lung tissues from mice were taken, treated with formalin, and subsequently embedded in paraffin and processed for sectioning. It was then deparaffinized to water, washed with antigen recovery, and blocked endogenous peroxidase for 10 min. CysLT1 antibody (AFFINITY, DF4865) was added and incubated overnight at 4°C. The next day, a biotinylated goat anti-rabbit IgG secondary antibody was added and incubated. Then horseradish enzyme-labeled affinity was added and incubated for 2 h. Color development was induced using DAB solution (SERVICEBIO, G1211) during a 10–30 min incubation period and then reacted with hematoxylin for 3 min at room temperature. Finally, they were monitored and photographed by a light microscope.

### 2.7. qPCR

Total RNA in lung tissue or cell was extracted with TRIzol reagent (vitality, B511311) after lung tissue was prepared into homogenates. PCR was performed for the measurement of differences in the mRNA expression. Then CDNA was reverse transcribed with the PrimeScript RT reagent kit (Takara, Japan) according to the manufacturer *s* instruction, and the CysLT1 gene level was detected with SYBR® Premix Ex Taq™ (Takara, RR820A) and real-time PCR instrument (Bio-Rad, USA, CFXConnect). The thermal cycling platform design was 95°C for 30 s, followed by 45 cycles of denaturation for 5 s at 95°C, an annealing step for 15 s at 60°C, and delay for 15 s at 72°C [23]. The expression of target genes was calculated by the 2^−−ΔΔCt^ method [24], and GAPDH was used as an internal reference. The primer sequence of the gene was shown in Table 1. Each sample was repeated three times to ensure the accuracy of the data.

### 2.8. Immunofluorescence Assay

Type II AEC cells were fixed with 4% paraformaldehyde. A total of 0.5% TritonX-100 was then added. Then we use gradient alcohol for dehydration and wash twice with distilled water. The section was blocked with 3% BSA for 30 min. Cells were incubated with primary antibody anti-*α*-SMA (cell signaling, 19245S) overnight at 4°C. Subsequently, the secondary antibody was added and incubated for 30 min. Then, it was washed with PBS (PH = 7.4) 3 times, 5 min each time. Then, the DAPI dye solution was dropped and incubated at room temperature avoiding light for 10 min. Quench tissues with a spontaneous fluorescence quench agent for 5 min. The tablets were then sealed with an anti-fluorescence quencher. Finally, the images were observed and collected under a fluorescence microscope.

### 2.9. Western Blot

Lung tissues and type II AEC cells were collected and lysed by a RIPA buffer (G2002, Servicebio, China). Then the total protein concentration was determined by a BCA kit (G2026, Servicebio, China). Protein samples were separated by electrophoresis on 10% SDS-PAGE gels before semidry transfer to PVDF membrane (10600023, GE Healthcare Life, USA) and then sealed with 5% BSA. The primary antibodies CysLT1 (affinity, DF4865) and *α*-SMA (affinity, AF1032) were added and incubated overnight at 4°C, followed by blocking with horseradish peroxidase-labeled goat anti-rabbit IgG secondary antibody blocking solution for 2 h at 4°C. GAPDH was used as loading controls. Protein bands were detected by ECL, and the protein gray value was calculated by ImageJ software.

### 2.10. Statistical Analysis

SPSS 20.0 statistical software was used for data analysis. One-way ANOVA analysis of variance was used for multiple groups of measurement data, and the Tukey test was used for comparison between groups. Kruskal–Wallis H test was used for variance. All data were expressed as mean ± standard deviation, and *P* < 0.05 indicated that the difference was statistically significant.

## 3. Results

### 3.1. BA Improved Histopathological Changes of Lung in Mice

The results of HE and Masson staining in the control group revealed that the bronchial structure was basically normal and clear; the airway epithelial cells were intact; and no proliferation, hypertrophy, and inflammatory cell infiltration were observed without blue collagen deposition (Figure 1(a)). Compared with the control group, there were lots of inflammatory cells infiltrated in the wall and alveolar interstitium in the IR group. The proliferation of airway epithelial cells was disordered, and mucous secretions were increased. Extensive blue collagen deposition and pulmonary fibrosis was evident. Relative to the IR group, the lung tissues in the IR + BA 50 mg/kg group were slightly improved, but the changes were not very obvious; the lung tissues in the IR + BA 100 mg/kg group were significantly improved, but there were still more inflammatory cell infiltrates; the lung tissues in the IR + BA 200 mg/kg group had basically returned to normal structures, without obvious damage and fibrosis.

Moreover, the semiquantitative scores of HE in Figure 1(b) declared that the IR group had evidently higher scores than that of the control group. While the semiquantitative scores of HE in IR + BA 100 mg/kg, IR + BA 200 mg/kg, and IR + DXM groups were extremely lower relative to the IR group. It was unveiled that BA ameliorated histopathological injury in mice.

### 3.2. BA Reduced the Levels of TGF-*β*, IL-1*β*, TNF-*α*, and IL-6 in Mice Serum

ELISA was used to detect the levels of TGF-*β*, IL-1*β*, TNF-*α*, and IL-6 in mice serum. The study found that the levels of TGF-*β*, TNF-*α*, IL-1*β*, and IL-6 in the IR group significantly increased than that in the control group (Figure 2). However, after giving BA and DXM, the contents of TGF-*β*, TNF-*α*, IL-1*β*, and IL-6 in the IR + BA 100 mg/kg, IR + BA 200 mg/kg, and IR + DXM groups significantly decreased than that in the IR group.

### 3.3. BA Reduced the Levels of CysLT, LTC4, and LTE4 in Mice BALF

As shown in Figure 3, relative to the control group, the levels of CysLT, LTC4, and LTE4 significantly increased in the IR group. However, administration of different concentrations of BA (50, 100, and 200 mg/kg) and DXM decreased the levels of CysLT, LTC4, and LTE4.

### 3.4. BA Reduced the Expression Level of CysLT1 in Mice Lung Tissue

The results of the immunohistochemical assay to determine the expression of CysLT1 in mice lung tissue were shown in Figure 4. The expression of CysLT1 significantly increased in the IR group than that in the control group. When treated with BA and DXM, it was found that the expression of CysLT1 in the IR + BA 50 mg/kg, IR + BA 100 mg/kg, IR + BA 200 mg/kg, and IR + DXM groups were lower than that in the IR group.

### 3.5. LTD4 Inhibited Viability of Type II AEC Cells, but BA Reversed the Inhibitory Effect

The effects of different concentrations of LTD4 and BA on the viability of type II AEC cells were detected by CCK8 assay, and the results were shown in Figure 5. Relative to the control group, the cell viability of type II AEC cells in the 37.5, 75, 150, and 300 nM LTD4 groups reduced (Figure 5(a)). Hence, 150 nM LTD4 was selected to establish the RILI cell model in type II AEC cells. Furthermore, given different concentrations of BA (20, 40, and 80 *μ*g/mL), it was found that BA reversed the LTD4-reduced type II AEC cell viability, and the higher the BA concentration, the more obvious the reversal effect (Figure 5(b)).

### 3.6. BA Reduced the Content of Collagen I Protein in LTD4-Induced Type II AEC Cells

The content of collagen I protein in type II AEC cells was detected by ELISA as shown in Figure 6. The result showed that the content of collagen I protein was significantly increased in the LTD4 group relative to the control group. However, after the administration of different concentrations of BA, it was found that BA reduced the content of collagen I protein in LTD4-induced type II AEC cells in a dose-dependent manner.

### 3.7. BA Reduced the Expression of *α*-SMA in LTD4-Induced Type II AEC Cells

The effect of BA on the level of *α*-SMA in LTD4-induced type II AEC cells was detected by immunofluorescence assay, and the results were shown in Figure 7. Relative to the control group, the expression of *α*-SMA was significantly increased in the LTD4 group. However, the expression of *α*-SMA was reversed after administration of different concentrations of BA.

### 3.8. BA Reduced the Expression of CysLT1 and *α*-SMA in RILI Lung Tissue and Type II AEC Cells

The CysLT1 mRNA levels in lung tissue and type II AEC cells were detected by qPCR. As shown in Figure 8(a), relative to the control group, the levels of CysLT1 mRNA in the IR and LTD4 groups increased, while the expression of CysLT1 mRNA decreased after treatment with different concentrations of BA. Moreover, the expressions of CysLT1 and *α*-SMA protein in lung tissue and type II AEC cells were detected by WB assay, the results were shown in Figures 8(b) and 8(c), indicating that the protein levels of CysLT1 and *α*-SMA were decreased *in vitro* and *in vivo* after BA treatment. In addition, it was further found that the addition of CysLT1 siRNA after LTD4/BA 80 treatment significantly reduced the expression of CysLT1 and *α*-SMA compared with LTD4+BA 80 *μ*g/mL group.

## 4. Discussion

RILI was a common complication of radiation therapy to a malignant tumor of the chest. RILI could develop into acute radiation pneumonitis, resulting in severe impairment of lung function and even death [25]. The treatment of RILI was often aimed at relieving pneumonia and pulmonary fibrosis [3]. BA was a flavonoid, which had a good effect on anti-inflammation and anti-fibrosis [17]. A mouse model of RILI was established by chest IR and a RILI cell model was established by LTD4 treatment of type II AEC cells to demonstrate that BA could ameliorate RILI through *in vivo* and *in vitro* experiments. Furthermore, further experimental results suggested that BA might attenuate RILI by inhibiting the CysLTs/CysLT1 signaling pathway.

Previous studies have found that IL-6, TNF-*α*, TGF-*β*, and IL-1*β* were elevated in lung inflammation [26, 27]. Zhang et al. found that BA could reduce the levels of IL-1*β*, IL-6, TNF-*α*, and inflammatory infiltration of lung tissue in BALF and improve the pathological changes in lung tissue [28]. This is consistent with the findings of this study that BA could improve the pathological tissue damage of RILI and reduce the levels of TGF-*β*, TNF-*α*, IL-6, and IL-1*β*. These mediators could promote EMT by activating fibroblasts and synthesizing extracellular matrix components such as type I collagen [29]. We examined the expression of type I collagen as well as the EMT marker *α*-SMA *in vitro* and *in vivo* and found that the higher concentrations of BA reduced the expression of type I collagen and *α*-SMA induced by IR or LTD4. This suppression effect on collagen I and *α*-SMA is in accordance with the report of Lu et al., which indicated a significant inhibitory effect of BA on pulmonary fibrosis in RILI [30].

Numerous studies have demonstrated that CysLTs were a kind of potent pro-inflammatory mediator in lung diseases, particularly pulmonary fibrosis and lung inflammation [31–33]. In pulmonary fibrotic diseases such as asthma, the production of inflammatory factors such as TGF-*β* and TNF-*α* usually tend to increase, which could promote the synthesis of CysLTs (CysLT, LTC4, and LTE4) [34]. This was similar to the levels of CysLTs, LTC4, and LTE4 increased in mouse lung tissue after IR stimulation in this study. After administration of BA, it could significantly reduce the levels of CysLTs, LTC4, and LTE4, and the expression of CysLTs immunohistochemistry. In addition, CCK8 experiments were performed, and it was found that LTD4 reduced the activity of type II ACE cells, which could be reversed by administration of baicalin. CysLTs/TP dual antagonists could inhibit nonacute pulmonary inflammation and also inhibit pulmonary fibrosis [35]. Therefore, the CysLTs/CysLT1 pathway played a vital role in pulmonary fibrosis and pulmonary inflammation.

CysLTs/CysLT1 pathway could alleviate RILI-induced pulmonary inflammation and fibrosis, and the regulatory effect of BA on CysLTs has been demonstrated [36]. Chung et al. explored the pharmacological effects of methanol extract of *Scutellaria baicalensis* Georgi root on gingival fibroblasts, found that flavonoids inhibited IL-1*β*-induced synthesis of LTB4, and could inhibit the lytic activity of collagen and enhance the cellular activity of fibroblasts [37]. Wu et al. reported that BA could inhibit the 5-Lox/CysLTs/CysLT inflammatory injury pathway by decreasing CysLTs content and inhibiting the expression of 5-Lox, CysLTs1, and CysLTs2 proteins [16]. This study found that BA could reduce CysLT1 mRNA level and the protein expression of CysLT1 and *α*-SMA *in vitro* and *in vivo*. These results suggested that BA could alleviate RILI by inhibiting the CysLTs/CysLT1 pathway.

However, this study also has some limitations. More proteins need to be detected in the specific mechanism of BA regulating the CysLTs/CysLT1 signaling pathway to prove the importance of the CysLTs/CysLT1 signaling pathway, so we will continue to do further research.

## 5. Conclusion

In conclusion, the study indicated that BA could ameliorate RILI by inhibiting the CysLTs/CysLT1 signaling pathway, thereby alleviating IR-induced pulmonary inflammation and pulmonary fibrosis. It further explained that BA might have a therapeutic effect on RILI.

## Figures and Tables

**Figure 1:** BA improved histopathological changes in the lung in mice. The results of HE staining (400-fold) and Masson staining (400-fold) in lung tissue of mice (a) and HE semiquantitative score (b). IR: irradiation, BA: baicalin, and DXM: dexamethasone. Compared with the control group, ^▲^*P* < 0.05 and ^▲▲^*P* < 0.01; compared with the IR group, ^#^*P* < 0.05 and ^##^*P* < 0.01. Data are expressed as the mean ± SD (*n* = 3) and were analyzed by one-way ANOVA followed by Tukey analysis.

**Figure 2:** BA reduced the contents of TGF-*β* (a), TNF-*α* (b), IL-1*β* (c), and IL-6 (d) in the serum of mice. IR: irradiation, BA: baicalin, and DXM: dexamethasone. Compared with the control group, ^▲^*P* < 0.05 and ^▲▲^*P* < 0.01; compared with the IR group, ^#^*P* < 0.05 and ^##^*P* < 0.01. Data are expressed as the mean ± SD (*n* = 6) and were analyzed by one-way ANOVA followed by Tukey analysis.

**Figure 3:** BA reduced the levels of CysLT (a), LTC4 (b), and LTE4 (c) in BALF of mice. IR: irradiation, BA: baicalin, and DXM: dexamethasone. Compared with the control group, ^▲^*P* < 0.05 and ^▲▲^*P* < 0.01; compared with the IR group, ^#^*P* < 0.05 and ^##^*P* < 0.01. Data are expressed as the mean ± SD (*n* = 6) and were analyzed by one-way ANOVA followed by Tukey analysis.

**Figure 4:** BA reduced the expression level of CysLT1 in the lung tissue of mice (400-fold). IR: irradiation, BA: baicalin, and DXM: dexamethasone. Compared with the control group, ^▲^*P* < 0.05 and ^▲▲^*P* < 0.01; compared with the IR group, ^#^*P* < 0.05 and ^##^*P* < 0.01. Data are expressed as the mean ± SD (*n* = 3) and were analyzed by one-way ANOVA followed by Tukey analysis.

**Figure 5:** LTD4 inhibited the viability of type II AEC cells, but BA reversed the inhibitory effect: (a) type II AEC cell viability decreased with increasing LTD4 concentration and (b) type II AEC cell viability increased with increasing BA concentration. Compared with the control or 0 *μ*g/mL group, ^▲^*P* < 0.05 and ^▲▲^*P* < 0.01. Data are expressed as the mean ± SD (*n* = 5) and were analyzed by one-way ANOVA followed by Tukey analysis.

**Figure 6:** BA reduced the content of collagen I protein in LTD4-induced type II AEC cells. LTD4: 150 nM LTD4-induced type II AEC cells and BA: baicalin. Compared with the control group, ^▲^*P* < 0.05 and ^▲▲^*P* < 0.01; compared with the LTD4 group, ^#^*P* < 0.05 and ^##^*P* < 0.01. Data are expressed as the mean ± SD (*n* = 6) and were analyzed by one-way ANOVA followed by Tukey analysis.

**Figure 7:** Immunofluorescence assay showed that BA reduced the expression of *α*-SMA in LTD4-induced type II AEC cells: (a) BA reduced the expression of *α*-SMA in LTD4-induced type II AEC cells (200-fold) and (b) BA reduced the fluorescence intensity of *α*-SMA in LTD4-induced type II AEC cells. LTD4: 150 nM LTD4-induced type II AEC cells and BA: baicalin. Compared with the control group, ^▲^*P* < 0.05 and ^▲▲^*P* < 0.01; compared with the LTD4 group, ^#^*P* < 0.05 and ^##^*P* < 0.01. Data are expressed as the mean ± SD (*n* = 3) and were analyzed by one-way ANOVA followed by Tukey analysis.

**Figure 8:** BA reduced the expression of CysLT1 mRNA, CysLT1, and *α*-SMA in lung tissue and type II AEC cells: (a) BA reduced the expression of CysLT1 mRNA in mice lung tissues and type II AEC cells and (b) and (c) BA reduced the expression of CysLT1 and *α*-SMA protein in mice lung tissues and type II AEC cells. IR: irradiation, BA: baicalin, DXM: dexamethasone, and LTD4: 150 nM LTD4-induced type II AEC cells. Compared with the control group, ^▲^*P* < 0.05 and ^▲▲^*P* < 0.01; compared with the IR or LTD4 group, ^#^*P* < 0.05 and ^##^*P* < 0.01; and compared with the LTD4 + BA 80 *μ*g/mL group, ^★^*P* < 0.05 and ^★★^*P* < 0.01. Data are expressed as the mean ± SD (*n* = 3) and were analyzed by one-way ANOVA followed by Tukey analysis.

**Table 1:** qPCR primer sequences.

Gene	Forward primer	Reverse primer
Mouse CysLT1	GACAGCCATGAGCTT TTTCC	ATGCACCCAGAGACA AGGTT
Mouse GAPDH	GACTCAACACGGGAAACCTCAC	CCAGACAAATCGCTCCACCAAC

## Data Availability

All data generated or analyzed during this study are included in this article.
